The article "Extraction, Chemical Composition, and Protective Effect of Essential Oil from Chimonanthus nitens Oliv. Leaves on Dextran Sodium Sulfate-Induced Colitis in Mice" was published in 2022. Journal: Oxid Med Cell Longev.

# Extraction, Chemical Composition, and Protective Effect of Essential Oil from *Chimonanthus nitens Oliv.* Leaves on Dextran Sodium Sulfate-Induced Colitis in Mice

**DOI:** 10.1155/2022/9701938

**Published:** 2022-07-06

**Authors:** Jing He, Yang Zhang, Kehui Ouyang, Lingli Chen, Wenya Meng, Ying Zhang, Wenjun Wang

**Affiliations:** ^1^Key Lab for Agro-Product Processing and Quality Control of Nanchang City, College of Food Science and Engineering, Jiangxi Agricultural University, Nanchang 330045, China; ^2^College of Animal Science and Technology, Jiangxi Agricultural University, Nanchang 330045, China

## Abstract

In this study, the essential oil (EO) was extracted by steam distillation from *Chimonanthus nitens Oliv*, and the extraction process was optimized by response surface methodology. The optimum process conditions are as follows: extraction time of 4.57 h, soaking time of 1.33 h, and solid-liquid ratio of 1 : 21.4. Under these conditions, the theoretical yield of EO is 1.5624%. The EO compounds were analyzed by gas chromatography-mass spectrometry (GC-MS). A total of 52 chemical components were detected, among which the content of 3-(4,8-dimethylnona-3,7-dienyl)-furan was the highest, accounting for 21.43% of the total peak area. The EO showed good antioxidant activity against 2,2-diphenyl-1-picrylhydrazyl (DPPH), 2,2′-azino-bis(3-ethylbenzthiazoline-6-sulfonic acid) (ABTS), and reducing power. In this study, we observed the protective effect of EO on ulcerative colitis (UC) induced by dextran sodium sulfate (DSS) in mice. EO effectively delayed weight loss and reduced DAI score. Histological examination also observed a significant reduction in damage in the EO group. The colon length of mice in DSS group was the shortest, and the colon length of mice in EO treatment group was longer than that in model group, but shorter than that in normal group (NOR : 8.17 ± 0.39 cm; DSS : 5.57 ± 0.93 cm; L − EO : 6.47 ± 0.78 cm; M − EO : 5.98 ± 0.58 cm; and H − EO : 6.1 ± 0.52 cm). The GSH activity in the L-EO and SASP groups was significantly higher than that in the DSS group (*P* < 0.01). SOD activity in L-EO and M-EO groups was also significantly higher than that in DSS treatment group (*P* < 0.01). MDA was decreased in the EO treatment groups and the SASP group (L-EO, H-EO, SASP: *P* < 0.01; M-EO: *P* < 0.05). MPO of EO treatment group was lower than that of model group (the L-EO group was not significant, M-EO: *P* < 0.05, H-EO: *P* < 0.05). This study shows that EO can effectively improve the symptoms of colitis.

## 1. Introduction

*Chimonanthus nitens Oliv* is a plant of the genus *Chimonanthus*, also known as edible herbal tea, golden tea in China [1]. It grows deep in the forests, and it is an important industrial crop [2]. *Chimonanthus nitens Oliv* is a nonfermented tea; it has been regarded as a natural food material of “medicine and food homology,” which is used to cool down the heat, strengthen the stomach, and treat abdominal distension and pain [3]. Studies have shown that *Chimonanthus nitens Oliv* has a good function of immune regulation, promoting digestion and reducing body fat [4, 5]. *Chimonanthus nitens Oliv* has an obvious fragrance and a high content of essential oil, which is one of the main active ingredients in *Chimonanthus nitens Oliv* [6]. Essential oil and other products are used in cosmetics and other industries. Previous studies have shown that *Chimonanthus nitens Oliv* essential oil has antioxidant and bacteriostatic ability [1]. In addition, essential oil also has anti-inflammatory activity [7].

The article "Extraction, Chemical Composition, and Protective Effect of Essential Oil from Chimonanthus nitens Oliv. Leaves on Dextran Sodium Sulfate-Induced Colitis in Mice" was published in 2022. Journal: Oxid Med Cell Longev.

Inflammatory bowel disease (IBD) is a chronic gastrointestinal disease with immune mechanism imbalance [8]. The pathogenesis of ulcerative colitis is caused by the interaction of multiple factors such as genetic factors, intestinal bacteria, and intestinal immune system disorders [9]. Colorectal cancer (CRC) is the most serious complication in patients with long-term ulcerative colitis. Clinical observation found that the mortality of patients with ulcerative colitis increased [10]. At the same time, ulcerative colitis-associated colorectal cancer (UC-CRC) exhibits unique clinicopathological features. In recent decades, foreign scholars have conducted a large number of clinical studies on UC-CRC. Foreign studies have reported that the incidence of cancer in ulcerative colitis patients with a course of 30 years is as high as 18%, and the overall risk of ulcerative colitis canceration is about 1.4% to 34% [11]. Because of differences in physical functions caused by geographical environment and ethnicity, the incidence of ulcerative colitis in Asia is lower than that in developed countries in Europe and America [12]. The lesion mainly occurred in the mucosa and submucosa from the colon to the rectum [13]. The main symptoms of patients include weight loss, decreased appetite, frequent abdominal pain, diarrhea, blood in the stool, and other conditions [14]. Traditional treatments for UC include anti-inflammatory drugs, steroids, immunomodulators, monoclonal antibodies, and antibiotic therapy, but most of these therapies have temporary effects, and there are serious complications and adverse drug reactions [15]. Studies have shown that many natural active substances have a good intervention effect on colitis, which can avoid the adverse effects brought by the traditional treatment of colitis [16]. Therefore, this study selected *Chimonanthus nitens Oliv* as raw material to explore the effect of its EO on colitis.

The article "Extraction, Chemical Composition, and Protective Effect of Essential Oil from Chimonanthus nitens Oliv. Leaves on Dextran Sodium Sulfate-Induced Colitis in Mice" was published in 2022. Journal: Oxid Med Cell Longev.

## 2. Materials and Methods

### 2.1. Chemicals and Regents

The *Chimonanthus nitens Oliv* leaves are purchased from Hunan, China; it is identified as *Chimonanthus nitens Oliv* by Professor Zhang Zhiyong (School of Agricultural Science, Jiangxi Agricultural University). The *Chimonanthus nitens Oliv* leaves collected in the experiment are in the mature stage. All materials are naturally dried. DSS (AR) was purchased from MP Biomedicals, USA. The detection kits for superoxide dismutase (SOD) (AR) were purchased from Jiancheng Institute of Biological Engineering (Nanjing, China).

### 2.2. Extraction of EO

EO extraction was done according to the methods of Kornbluth [17]. Place *Chimonanthus nitens Oliv* leaf powder (40.0 g) into a beaker; a certain amount of distilled water (material vs. water =1 : 15-1 : 25) was added into the beaker to soak, all of which was then transferred to a 2000 mL distillation flask. The sample was distilled with steam by the Clevenger apparatus. The water fraction containing EO drops into the phase separation tube. After heating for a period of time (3-5 h), the EO was collected and dried overnight on anhydrous sodium sulfate. Finally, the obtained EO was stored at 4°C. The yield of essential oil is calculated as follows [18]:

(1) $$\begin{array}{c} Y\left(\%\right)=\frac{m}{M}\times 100, \end{array}$$

where *Y* (mL/g) represents the yield of EO, *m* (g) represents the quality of the obtained EO, and *M* (g) represents the quality of the raw material sample.

### 2.3. BBD for EO Extraction

So as to obtain the best extraction conditions of EO, the response surface optimization design of three factors and three levels was designed to investigate the individual and interactive effects of process variables according to the results of single factor tests and the principle of Box-Behnken combination test design [19]. The three independent variables were extraction time (*X*_1_: 3-5 h), soaking time (*X*_2_: 0-2 h), and material-to-liquid ratio (*X*_3_: 1 : 15-1 : 25), while the yield of EO (*Y*) was selected as the dependent variable. The temperature was fixed at 120°C.  Table 1 shows the different permutations of the response surface tests with a total of 17 different combinations; each combination is extracted repeatedly three times, including five replicates at the center point to fit the complete second-order polynomial equation model. The basic data of three factors and three levels in the response surface design is 12 groups. The reason why there are more than 12 groups is that it is necessary to do a center point repeat test to investigate the fit of the center area, and the number of repeat groups is required to be no less than 3 times. To avoid waste, the number of repetitions should not be too much. The default number of times of the software is 5 times. Based on the above factors, 5 repeated experiments were selected. In the end, there are 17 combinations in total. In formula (2), where *Y* is the predicted EO yield, *β*_0_ is a constant, *β*_*i*_, *β*_*ii*_, and *β*_*ij*_ are the regression coefficients for linearity, quadratic, and the interaction coefficient between the three factors, while *X*_*i*_ and *X*_*j*_ are levels of the independent variables and *ε* is the residual associated to the experimental [20].

(2) $$\begin{array}{c} Y=\beta_{0}+\overset{3}{\underset{i=1}{\sum }}\beta_{i}X_{i}^{2}+\overset{3}{\underset{i=1}{\sum }}\beta_{ii}X_{i}^{2}+\overset{3}{\underset{i=1}{\sum }}\overset{3}{\underset{j=i+1}{\sum }}\beta_{ij}X_{i}X_{j}+\varepsilon . \end{array}$$

In order to reflect the characteristics of the response surface more intuitively, the regression coefficient is applied to model fitting and the response surface is generated on the three-dimensional curve and contour map. The independent variables were coded as -1 (low value), 0 (center point), and +1 (high value). The related mathematical equations were as follows [21]:

(3) $$\begin{array}{c} X=\frac{X_{i}-X_{0}}{\Delta X_{i}}, \end{array}$$

where *X* is the coded value of *X*_*i*_, *X*_0_ is the value of independent variable at the center point, and Δ*X*_*i*_ is the step change.

The article "Extraction, Chemical Composition, and Protective Effect of Essential Oil from Chimonanthus nitens Oliv. Leaves on Dextran Sodium Sulfate-Induced Colitis in Mice" was published in 2022. Journal: Oxid Med Cell Longev.

### 2.4. GC-MS Analysis

The composition of EO was determined by GC-MS according to Guadalupe's methods described previously [22]. The GC-MS analyses were performed with an Agilent model 7890B gas chromatograph (Agilent Technologies Inc., USA) coupled to an Agilent 5977A Mass Spectrometry (Agilent Technologies Inc., USA). The EO was separated on a HP-5MS quartz capillary column (30 m × 0.25 *μ*m × 0.25 *μ*m) with high-purity helium as carrier gas at a flow rate of 1.0 mL/min and a split ratio of 1 : 10. The injector temperature was set at 250°C, and the column furnace temperature was kept at 40°C for 5 min, then increased to 170°C at 3°C/min for 5 min, and then increased to 280°C at 10°C/min for 5 min.

The mass spectrometry scanning conditions are as follows: EI is the ionization source, the ionization energy is 70 eV, the ion trap temperature is 200°C, the manifold temperature is 40°C, the transmission line temperature is 250°C, and the mass scanning range is 40-480 amu.

### 2.5. Antioxidant Activities

The DPPH radical scavenging method, ABTS method, and reducing power method were used to determine the antioxidant capacity of EO. With ascorbic acid as reference, the antioxidant capacity of EO was compared.

The article "Extraction, Chemical Composition, and Protective Effect of Essential Oil from Chimonanthus nitens Oliv. Leaves on Dextran Sodium Sulfate-Induced Colitis in Mice" was published in 2022. Journal: Oxid Med Cell Longev.

#### 2.5.1. DPPH Assay

The DPPH radical scavenging effect of EO was established by previous methods [23]. Briefly, different concentrations of EO alcohol solution were mixed with DPPH solution (0.1 mM), and the absorbance value was measured at 517 nm after 30 min of reaction at 37°C: Vc (ascorbic acid) as a positive control. The instrument used is the Thermo microplate reader (Multiskan, USA). The clearance rate of DPPH free radical was calculated by the following formula:

(4) $$\begin{array}{c} \%\text{inhibition}=\left[100*\left(\frac{{\text{Abs}}_{\text{control}}–{\text{Abs}}_{\text{sample}}}{{\text{Abs}}_{\text{control}}}\right)\right], \end{array}$$

where Abs_control_ represents the absorbance value of blank control group and Abs_sample_ represents the absorbance value of the sample group.

#### 2.5.2. ABTS Assay

The antioxidant capacity of EO can be assessed by the ABTS method [24]. ABTS free radical cations were prepared by reaction of ABTS solution of 7 mM with ammonium persulfate of 2.45 mM. The mixture was kept in the darkness at 37°C for 16 h. Then, the radical solution was diluted with methanol to obtain an absorbance of 0.70 ± 0.02 at 734 nm. The EO solutions of different concentrations were mixed with ABTS, and the absorbance was measured at 743 nm: Vc as a positive control. The instrument used is the Thermo microplate reader (Multiskan, USA). The ABTS free radical inhibition rate is calculated as follows:

(5) $$\begin{array}{c} \%\text{inhibition}=\left[100*\left(\frac{{\text{Abs}}_{\text{control}}–{\text{Abs}}_{\text{sample}}}{{\text{Abs}}_{\text{control}}}\right)\right], \end{array}$$

where Abs_control_ represents the absorbance value of blank control group and Abs_sample_ represents the absorbance value of the sample group.

#### 2.5.3. Reduction Capability Assay

The method of measuring the reducing power capacity of EO was improved on the basis of previous methods [25]. The EO alcohol solutions of different concentrations were mixed with 0.2 mL phosphate-buffered solution (pH 6.6) and potassium ferricyanide solution (2.5 mL 1%). The mixture was bathed in water at 50°C for 20 min, then added 2.5 mL trichloroacetic acid solution (10%, *V*/*W*), and centrifuged at 3000 r/min for 10 min. The supernatant (2.5 mL) was transferred into a test tube; ferric chloride solution (0.5 mL 0.1%) and distilled (2.5 mL) water were added. The absorbance value was read at 700 nm.

### 2.6. Experimental Animals and Grouping

A total of 66 wild-type SPF male BALB/c mice aged 6-8 weeks (18-20 g) were purchased from Hunan Slack Jingda Animal Experiment Co., Ltd. (Hunan, China). During the experiment, the mice were housed in a 12 h day/night cycle environment with room temperature of 23 ± 2°C and humidity of 55 ± 5%, with access to feed and water *ad libtum*. There was adaptive feeding for one week before the trial began. All the experiments were carried out strictly in accordance with the Guide for the Care and Use of Laboratory Animals of the Chinese Association for Laboratory Animal Science and approved by the Animal Care and Use Committee of the Jiangxi Agricultural University (JXAUA01).

The article "Extraction, Chemical Composition, and Protective Effect of Essential Oil from Chimonanthus nitens Oliv. Leaves on Dextran Sodium Sulfate-Induced Colitis in Mice" was published in 2022. Journal: Oxid Med Cell Longev.

According to the method of Trivedi and Jena [26], sixty-six mice were randomly divided into 6 groups with 11 mice in each group: blank control group (Normal), DSS group (DSS), positive treatment group (SASP (sulfasalazine) 200 mg/kg), high-dose treatment group (H-EO 200 mg/kg), medium-dose treatment group (M-EO 100 mg/kg), and low-dose treatment group (L-EO 50 mg/kg). EO was administered to mice by gavage. During the experiment, except for the blank control group, 3% DSS (*W*/*V*) was given to the other experimental groups to induce ulcerative colitis, which was freely drunk for 9 consecutive days, and fresh DSS solution was replaced every two days.

### 2.7. Evaluation of Disease Activity Index (DAI) and Sample Collection

Body weight, fecal character, and bleeding conditions were recorded every day during the experiment. DAI was recorded according to the existing scoring criteria [DAI = (weight loss score + stool characters score + hematochezia score)/3] [27]. On day 10, blood was collected from the eyes of all mice, centrifuged at 3000 r/min for 10 min, and the supernatants were stored at -80°C for further analysis as soon as possible. Colons of mice in each group were collected, and their lengths were measured, and fresh colonic tissues were separated from the distal large intestine for histological analysis.

### 2.8. Histopathological Examination of the Colon

The colon was fixed in 4% paraformaldehyde, dehydrated, and transparentized. After paraffin embedding, the colon was selected, dewaxed and stained with HE, transparentized and sealed, and observed under an upright microscope (Nikon Japan), and the histopathological scoring standard was in accordance with Murano standard: degree of inflammatory infiltration (0-5), degree of crypt injury (0-4), degree of ulcer (0-3), and whether there is edema (0 or 1) .

### 2.9. Biochemical Index Detection

Colon tissues of mice in each group were taken, and lysis buffer was added. The mixture was homogenized in a tissue homogenizer and centrifuged at 3000 r/min for 10 min. The supernatant after centrifugation was collected and stored at -80°C for subsequent tests. Total protein content was determined with BCA protein detection kit. The activities of myeloperoxidase (MPO), SOD, MDA, and GSH-PX in colon tissue and serum were determined by kit according to the manufacturer's instructions.

The article "Extraction, Chemical Composition, and Protective Effect of Essential Oil from Chimonanthus nitens Oliv. Leaves on Dextran Sodium Sulfate-Induced Colitis in Mice" was published in 2022. Journal: Oxid Med Cell Longev.

### 2.10. Statistical Analysis

The software used in response surface design is design expert 8.0. All data were expressed as the mean ± SD (standard deviation) using SPSS statistical software (version 22.0, IBM, Armonk, NY, USA). Duncan's test was used to evaluate the differences between groups. *P* < 0.05 means statistically significant difference.

## 3. Results and Discussion

### 3.1. Optimization of Extraction Process of EO by Steam Distillation

#### 3.1.1. Fitting the Response Surface Model

The response surface experiment design is shown in Table 1. In addition, multiple regression analysis technology was used to analyze the reliability of the regression equation of the model, and the results are shown in Table 2. The quadratic polynomial equation is expressed as

(6) $$\begin{array}{c} Y=1.55+0.028*X_{1}+0.022*X_{2}+0.009*X_{3}+0.002*X_{1}X_{2}-0.003*X_{1}X_{3}-0.001*X_{2}X_{3}-0.015*{X_{1}}^{2}-0.038*{X_{2}}^{2}-0.052*{X_{3}}^{2}, \end{array}$$

where *Y* extraction yield of *Chimonanthus nitens Oliv* leaf EO (expressed in g per 100 g of dry weight) (%), *X*_1_ extraction time (h); *X*_2_ soaking time (h); and *X*_3_ plant material to water ratio (g: mL).

The quadratic model showed that *X*_1_ − *X*_3_ and *X*_1_*X*_2_ had a good effect on the extraction rate, while the quadratic variables *X*_1_^2^ − *X*_3_^2^ and the variable interactions *X*_1_*X*_3_ and *X*_2_*X*_3_ showed negative effects.

#### 3.1.2. Analysis of Variance (ANOVA) Evaluation

As shown in Figure 1(a), the data in the normal % probability graph is a straight line, indicating that the model is sufficient and there is no variance bias in the data.  Figure 1(b) shows that the predicted values of the model are in good agreement with the experimental data [28]. All points in the internal residual plot are within the limit (±3), indicating good model adequacy (Figure 1(c)).

As can be seen from Table 2, the model is significant; *F* value is 48.81 (*P* < 0.0001), indicating a good fitting and prediction for the experimental data [29]. The model is also tested by an *F* test [30]. Lack-of-fit is an indicator to measure the degree of fitting between model and data. According to the results in Table 2, the lack-of-fit with the *P* value (0.61) is greater than 0.05 (not significant), indicating that the prediction model reasonably represents the observed value, which means that the model is accurate enough to predict the relevant response. The coefficient of variation (CV) describes the degree of dispersion of the data. Coefficient of variation (CV) was 0.56%, indicating small variation and high repeatability [31]. The regression model predicted that the coefficient of determination *R*^2^ for the extraction rate was 0.9843, which meant that 98.43% of the sample variation could be attributed to the independent variable and the model could not explain 1.57% of the total variation; thus, the fitting of regression model is in good agreement with experimental data [32]. Meanwhile, the adjusted approximation values of *R*^2^ (0.9641) and *R*^2^ (0.9843) confirmed the good model sufficiency and the strong correlation between the predicted value and the experimental value.

The article "Extraction, Chemical Composition, and Protective Effect of Essential Oil from Chimonanthus nitens Oliv. Leaves on Dextran Sodium Sulfate-Induced Colitis in Mice" was published in 2022. Journal: Oxid Med Cell Longev.

#### 3.1.3. Analysis of Response Surfaces

Elliptic contour lines indicate significant interactions between variables, while circular contour lines indicate insignificant interactions between variables.  Figure 2 depicts the interaction between distillation time and immersion time on the extraction rate of EO. The extraction rate of EO increased with the extension of extraction time [33]. However, when the extraction time increased to a certain extent, the yield of EO did not increase significantly. This is due to the decrease of extraction rate due to the volatilization of some volatile substances with the extension of heating time.

As can be seen from Figure 2, the extraction rate of EO gradually increases with the increase of solid-liquid ratio. Our results are consistent with previous literature reports on steam distillation and steam distillation of other plant essential oils (S. [34, 35]). In the steam distillation process, the role of water is to prevent the thermal degradation of substances. Although a large amount of solvent can obtain a high extraction rate, it can also lead to the extraction process is difficult and unnecessary waste of solvent. If the amount of solvent is small, the extraction will be incomplete. Therefore, choosing the right liquid-solid ratio is very important. With the increase of liquid-solid ratio, the yield of EO increased [36].

According to the response surface shown in Figure 2, the extraction rate of EO was also closely related to the soaking time. With the increase of the soaking time and the solid-liquid ratio, the yield of EO gradually increased at first and then gradually decreased after increasing to a certain value [37]. This phenomenon is attributed to the fact that soaking the material in water facilitates cell expansion and dissolution of intracellular components.

All the factors had positive effects on the extraction rate of EO. The steep curvature in extraction time, soaking time, and solid-liquid ratio showed that the extraction rate of EO responded very quickly to these factors. The order of positive influence was extraction time, soaking time, and solid-liquid ratio. On the basis of BBD optimization, the optimum conditions of extraction time of 4.57 h, solid-liquid ratio of 1 : 21.4, soaking time of 1.33 h were obtained. Under these conditions, the theoretical yield of EO is 1.5624%.

The article "Extraction, Chemical Composition, and Protective Effect of Essential Oil from Chimonanthus nitens Oliv. Leaves on Dextran Sodium Sulfate-Induced Colitis in Mice" was published in 2022. Journal: Oxid Med Cell Longev.

#### 3.1.4. Verification Experiments

In order to verify the accuracy of the optimization conditions, the extraction time, soaking time, and solid-liquid ratio were adjusted to 4.57 h, 1.33 h, and 1 : 21.4. After three parallel experiments, the actual yield of EO is 1.5592 ± 0.03%. The highest yield is observed in Table 1: when the extraction time, soaking time, and solid-liquid ratio are 4 h, 1 h, and 1 : 20, respectively, the yield of EO is 1.562%. On the basis of BBD optimization, the optimum conditions of extraction time (4.57 h), solid-liquid ratio (1 : 21.4), and soaking time (1.33 h) were obtained. Under these conditions, the predicted theoretical yield of EO is 1.5624%. The actual yield of EO is 1.5592 ± 0.03%. The values are observed in Table 1; the experimental predicted values and the experimental actual values are very similar, indicating that the design of BBD is reliable.

### 3.2. Chemical Composition of EO

Under the optimum conditions, the EO compounds were analyzed by gas chromatography-mass spectrometry. *Chimonanthus nitens Oliv* EO is a transparent pale yellow liquid with a unique fragrance. The composition analysis of EO is shown in Figure 3 and Table 3. A total of 52 chemical components were detected, among which the content of 3-(4,8-Dimethylnona-3,7-dienyl)-furan was the highest, accounting for 21.43% of the total peak area, followed by camphor (11.85%) and long leaf aldehyde (10.51%). The compounds in EO mainly contain alkanes, alcohol, and esters. The types of terpenes detected in this work are similar to the results of Giampieri [38].

### 3.3. Antioxidant Activity Analysis *In Vitro*

The antioxidant activity of plant essential oils is a complex process occurring through different mechanisms, so the free radical scavenging ability of plant EO needs to be realized by a variety of *in vitro* tests. Therefore, ABTS, DPPH, and reducing power method were used to test the antioxidant capacity of *Chimonanthus nitens Oliv* EO.

The DPPH free radical scavenging model is often used to evaluate the antioxidant properties of compounds [39, 40]. As shown in Figure 4, the concentration of EO was 2-10 mg/mL, the scavenging ability of DPPH was 15%-41%, and free radical scavenging activity was positively correlated with EO concentration. The antioxidant capacity of EO is expressed by IC_50_ value (the scavenging rate can reach 50% of the EO concentration). The results showed that the DPPH radical scavenging rate reached 50% when the concentration of EO was 14.6 mg/mL. The *Chimonanthus nitens Oliv* EO showed stronger DPPH scavenging activity. The abundance of oxy sesquiterpenes in the EO of Paramignya lobata was low, with IC50 of 82.4 mg/mL [41].

The article "Extraction, Chemical Composition, and Protective Effect of Essential Oil from Chimonanthus nitens Oliv. Leaves on Dextran Sodium Sulfate-Induced Colitis in Mice" was published in 2022. Journal: Oxid Med Cell Longev.

After being oxidized in the reaction system, ABTS will generate a stable free radical, which is blue-green and has characteristic absorption at 734 nm. The addition of free radical scavenger will weaken the color and reduce the absorbance. The degree of decrease reflects its ability to scavenge free radicals [42, 43]. The scavenging ability of EO on ABTS free radicals is shown in Figure 4. Both EO and Vc have good scavenging effect on ABTS free radicals, and the scavenging rate increases with the increase of EO. When the concentration of EO reached 10 mg/mL, the clearance rate reached 94%.

There is a great correlation between reducing power and oxidation resistance. The absorption value is positively correlated with reducing force [44]. As shown in Figure 4, both EO and Vc have good reducing power. The reducing power of the two increased significantly between the concentrations of 2 and 150 mg/mL; the reducing power increased with the increase of EO concentration.

### 3.4. Intervention of EO on Ulcerative Colitis in Mice

Plant EO mainly contains small molecule aldehydes, esters, monoterpenes, sesquiterpenes, and small molecule aromatic compounds [45]. Studies have shown that amomum EO is mainly monoterpenoids and sesquiterpenoids. EO with a content of more than 1% are camphor acetate, camphor, limonene, camphor hydrocarbons, borneol, *β*-pinene, *β*-myrcene, and *α*-pinene. Amomum EO can improve colonic mucosal inflammation in TNBS-induced colitis rats [46]. Wang et al. found that the main constituents of lavender EO are linalool, linalyl acetate, eucalyptol, B-ocimenes (both cis and trans), terpene-4-ols, and camphor. The EO has a protective effect on mice with ulcerative colitis caused by DSS [47]. The EO of *Chimonanthus nitens Oliv* also contains D-camphor, bornyl isovalerate, neryl acetate, pinene, myrcene, etc. It shows that these compounds in EO have a protective effect on colitis mice. Therefore, this experiment explored the protective effect of *Chimonanthus nitens Oliv* EO on DSS-induced ulcerative colitis.

In this study, DSS-induced mice developed significant symptoms of colitis, including drowsiness, weight loss, diarrhea, and fecal bleeding, compared to the control group. Compared with the DSS group, EO effectively delayed weight loss (Figure 5) and reduced DAI score (Figure 5). This is consistent with the findings of Li et al. [48]. The overall symptoms of mice in the DSS group were cecal atrophy and colonic shortening. The intervention of EO significantly restored the shortening of colon length induced by DSS in a dose-dependent manner. The animals showed signs of softening feces 4 days after taking the drug. After 6 days, the body weight of mice in the DSS group was significantly lower than that in the control group (Figure 5, *P* < 0.01). Histological examination also observed a significant reduction in damage in the EO group (Figure 6). These results indicated that EO had an inhibitory effect on colitis.

The article "Extraction, Chemical Composition, and Protective Effect of Essential Oil from Chimonanthus nitens Oliv. Leaves on Dextran Sodium Sulfate-Induced Colitis in Mice" was published in 2022. Journal: Oxid Med Cell Longev.

### 3.5. Effect of Essential Oils on Histological Changes

Colonic length is another indicator to reflect the severity of intestinal inflammation [49]. As shown in Figure 7, the colon length of mice in the DSS group was the shortest, and the colon length of mice in the EO treatment group was longer than that in model group, but shorter than that in normal group (NOR: 8.17 ± 0.39 cm; DSS: 5.57 ± 0.93 cm; L-EO: 6.47 ± 0.78 cm; M-EO: 5.98 ± 0.58 cm; and H-EO: 6.1 ± 0.52 cm). The more severe the inflammation of colitis, the shorter is the length of the colon [50]. Shortening of the colon is one of the typical symptoms of colitis. [51].

As shown in Figure 6, the epithelium in colon tissue sections of mice in the normal group was intact, while crypt glands, stroma, and submucosal structures were not damaged. In the DSS model group, inflammatory cells were infiltrated in the submucosa and muscularis, the mucosa lamina propria had the most severe erosion, crypt structure was deformed or disappeared, and intestinal cells were lost. The positive group and the EO dose group could reduce the damage of colon epithelia caused by DSS, also could inhibit inflammatory cell infiltration, and could maintain the integrity of intestinal epithelia and crypt glands. Huang et al. found similar results [52]. The histological score of mice in DSS group was significantly higher than that in normal group (*P* < 0.01). Clearly, essential oils have reversed this upward trend. The significance of groups L-EO, M-EO, H-EO, and SASP was lower than that of DSS group (*P* < 0.01). Li et al. also found that cinnamon essential oil could significantly reduce colon tissue damage caused by DSS [48].

### 3.6. Essential Oil of *Chimonanthus nitens Oliv* Improves Colonic Oxidation Index

Invasion of colon tissue by immune cells is a typical event of colitis [53]. Local inflammatory reaction can cause lipid peroxidation of unsaturated fatty acids on the biofilm, thus leading to oxidative stress damage of the tissue [51, 54]. Malondialdehyde (MDA) is one of the important indicators of oxidative stress in the body [55]. In addition, the activity of GSH-PX and SOD can also reflect the antioxidant capacity of the body [56]. MPO activity is one of the important biomarkers of neutrophil infiltration (X. [57]). As shown in Figure 8, MDA in colon of mice treated with DSS was significantly higher than that in normal group (*P* < 0.01). MDA was decreased in the essential oil treatment groups and the SASP group (L-EO, H-EO, SASP: *P* < 0.01, M-EO: *P* < 0.05). Compared with the normal group, the colon GSH-PX and SOD activities of mice after DSS intervention were significantly decreased (*P* < 0.01, *P* < 0.05). The activity of GSH-PX and SOD in colon tissue was increased in different degrees after treatment with different doses of EO. The GSH activity in the L-EO and SASP groups was significantly higher than that in the DSS group (*P* < 0.01). SOD activity in L-EO and M-EO groups was also significantly higher than that in DSS treatment group (*P* < 0.01). MPO enzymes in the model group were significantly higher than those in the control group (*P* < 0.01). The EO treatment group was lower than the model group (the L-EO group was not significant, M-EO: *P* < 0.05, H-EO: *P* < 0.05). This result is similar to Li's discovery [58].

The article "Extraction, Chemical Composition, and Protective Effect of Essential Oil from Chimonanthus nitens Oliv. Leaves on Dextran Sodium Sulfate-Induced Colitis in Mice" was published in 2022. Journal: Oxid Med Cell Longev.

## 4. Conclusions

In this study, the EO of *Chimonanthus nitens Oliv* was extracted by steam distillation, and the extraction process was investigated and the optimal extraction conditions were obtained by response surface methodology: extraction time of 4.57 h, soaking time of 1.33 h, and solid-liquid ratio of 1 : 21.4. The yield of EO is 1.5624%. The extraction time had the greatest effect on the yield of EO, followed by soaking time and solid-liquid ratio. The constituents of the EO were analyzed by GC-MS. A total of 52 constituents were identified, of which 3-(4,8-dimethylnona-3,7-dienyl)-furan was the highest, accounting for 21.43%. The EO showed good antioxidant activity and scavenging effect on free radicals. Therefore, the effect of EO on DSS induced colitis in mice was explored, and the results showed that the treatment of EO dose group could reduce the colon injury caused by DSS. However, the specific mechanism needs to be further explored.

## Figures and Tables

**Figure 1:** Diagnostic plots of model adequacy. Normal % probability (a), predicted versus actual (b), and internally studentized residuals (c).

**Figure 2:** Response surface and contour plots for the effect of independent variables on extraction yield of essential oil.

**Figure 3:** Total ion flow chromatography of EO.

**Figure 4:** Scavenging activities of EO on DPPH radical, ABTS radical, and reducing power in vitro. VC (vitamin C) was used as positive control; ^∗∗^*P* < 0.01, versus VC at the same concentration.

The article "Extraction, Chemical Composition, and Protective Effect of Essential Oil from Chimonanthus nitens Oliv. Leaves on Dextran Sodium Sulfate-Induced Colitis in Mice" was published in 2022. Journal: Oxid Med Cell Longev.

**Figure 5:** The daily body weight changes and the disease activity index (DAI) in mice.

**Figure 6:** The representative photographs of H&E staining (magnification: ×200) and scores of colonic mucosa of mice. ^∗^*P* < 0.05 and^∗∗^*P* < 0.01 vs. normal control; ^#^*P* < 0.05 and^##^*P* < 0.01 vs. the DSS group.

**Figure 7:** Effects of EO on the colon length of colitis in mice. ^∗^*P* < 0.05 and^∗∗^*P* < 0.01 vs. normal control; ^#^*P* < 0.05 and^##^*P* < 0.01 vs. the DSS group.

**Figure 8:** Effects of EO on the levels of MPO, MDA, GSH and SOD in colon tissue of colitis mice. ^∗^*P* < 0.05 and^∗∗^*P* < 0.01 vs. normal control; ^#^*P* < 0.05 and^##^*P* < 0.01 vs. the DSS group.

**Table 1:** Results of the BBD design for the extraction of essential oil from *Chimonanthus nitens Oliv*.

Run	Extraction time (h)	Soaking time (h)	Material-to-liquid ratio	The yield of EO (%)
	*X*_1_	*X*_2_	*X*_3_	*Y*
1	3	0	1 : 20	1.45
2	5	0	1 : 20	1.508
3	3	2	1 : 20	1.485
4	5	2	1 : 20	1.55
5	3	1	1 : 15	1.45
6	5	1	1 : 15	1.505
7	3	1	1 : 25	1.47
8	5	1	1 : 25	1.513
9	4	0	1 : 15	1.425
10	4	2	1 : 15	1.475
11	4	0	1 : 25	1.45
12	4	2	1 : 25	1.495
13	4	1	1 : 20	1.56
14	4	1	1 : 20	1.55
15	4	1	1 : 20	1.562
16	4	1	1 : 20	1.547
17	4	1	1 : 20	1.54

**Table 2:** ANOVA of response surface quadratic model for extraction yield of essential oil from *Chimonanthus nitens Oliv*.

Variables	Sun of squares	df	Mean square	*F* value	*P* value	
Model	0.031	9	0.003427	48.81	<0.0001	Significant
*X*_1_	0.006105	1	0.006105	86.94	<0.0001	
*X*_2_	0.003698	1	0.003698	52.66	0.0002	
*X*_3_	0.0006661	1	0.0006661	9.49	0.0178	
*X*_1_ *X*_2_	0.00001225	1	0.00001225	0.17	0.6887	
*X*_1_ *X*_3_	0.000036	1	0.000036	0.51	0.4972	
*X*_2_ *X*_3_	0.00000625	1	0.00000625	0.089	0.7741	
*X*_1_^2^	0.0009664	1	0.0009664	13.76	0.0076	
*X*_2_^2^	0.006209	1	0.006209	88.42	<0.0001	
*X*_3_^2^	0.011	1	0.011	163.07	<0.0001	
Residual	0.0004916	7	0.00007022			
Lack of fit	0.0001548	3	0.00005158	0.61	0.6418	Not significant
Pure error	0.0003368	4	0.0000842			
*R* ^2^	0.9843					
Adj *R*^2^	0.9641					
C.V. %	0.56					
Adep precision	19.048					
Cor total	0.031	16				

**Table 3:** Composition and content of *Chimonanthus nitens Oliv* essential oil.

Peak	Compound	CAS number	RT	Area (%)
1	3-Carene	13466-78-9	4.643	0.61
2	Camphene	79-92-5	4.974	2.08
3	(1-Methylethyl)-4-methylene-Bicyclo[3.1.0]hexane	3387-41-5	5.595	0.15
4	(1S)-(1)-*β*-Pinene	18172-67-3	5.825	0.27
5	D-Limonene	5989-27-5	6.974	0.30
6	Eucalyptol	470-82-6	7.100	4.8
7	Terpinolene	586-62-9	9.010	0.13
8	(+)-2-Bornanone	464-49-3	11.566	11.85
9	(1R,2R,5R,E)-7-Ethylidene-1,2,8,8-tetramethylbicyclo[3.2.1]octane	193695-14-6	18.073	0.43
10	L-Bornyl acetate	5655-61-8	18.539	3.45
11	Terpineol	93836-50-1	20.164	0.65
12	(-)-*β*-Elemene	20307-84-0	21.932	5.21
13	Copaene	3856-25-5	23.120	0.75
14	*cis*-3,7-Dimethyl-2,6-octadien-1-yl acetate	141-12-8	23.629	0.48
15	Bicyclosesquiphellandrene	54274-73-6	23.836	1.71
16	*β*-Elemene	515-13-9	23.946	0.38
17	4,8,8-Trimethyl-2-methylene-4-vinylbicyclo[5.2.0]nonane	242794-76-9	25.227	2.27
18	*α*-Bergamotene	18252-46-5	26.026	0.24
19	Hexahydronaphthalene	267665-20-3	26.715	0.5
20	Tetramethyl-cycloundecatriene	1000062-61-9	26.869	1.17
21	*cis*-*β*-Farnesene	28973-97-9	27.164	0.32
22	*δ*-Cadinene	483-76-1	27.936	5.69
23	*γ*-Cadinene	39029-41-9	28.106	0.5
24	Methylenetricyclo-decane	18252-44-3	28.319	1.00
25	Aciphyllene	87745-31-1	28.571	0.11
26	Cyperene	2387-78-2	29.069	0.25
27	*β*-Bergamotene	1000425-19-8	29.249	0.18
28	Hexahydro dimethyl naphthalene	17627-24-6	29.457	1.65
29	Bornyl isovalerate	76-50-6	29.704	0.3
30	Dimethyl octahydro naphthalene	123123-37-5	30.306	0.54
31	Cubenene	29837-12-5	31.232	0.55
32	Butadienyl dimethyl octane	1000195-92-1	31.532	0.62
33	Peroxydiene	1000140-33-3	31.910	0.93
34	*β*-Oplopenone	28305-60-4	33.136	2.22
35	Longifolenaldehyde	19890-84-7	33.360	10.51
36	3-(4,8-Dimethylnona-3,7-dienyl)-furan	23262-34-2	34.214	21.43
37	Neoclovene oxide	1000163-73-4	35.194	3.6
38	2-Heptanone	90165-09-6	36.513	0.14
39	(+)-Epicubenol methylethyl	19912-67-5	38.762	0.36
40	Isoaromadendrene epoxide	1000159-36-6	40.366	0.88
41	4-Hexen-1-ol	1000221-57-6	40.618	0.37
42	Tetramethyl-hexahydro-Benzopyran	41678-32-4	41.017	0.14
43	Dimethyl-2,3-diethenyl-1,5-cyclohexane	74806-57-8	41.636	0.17
44	1-adamantyl methyl ester	1000282-92-0	42.358	0.74
45	Dimethylspiro cyclooctane	77143-32-9	44.586	0.13
46	Costol	515-20-8	45.878	0.12
47	*α*-Santalyl palmitate	1000465-97-2	47.925	0.72
48	Dimethyl cyclohexane	74806-56-7	49.715	0.61
49	Farnesol isomer	1000108-92-4	49.977	0.14
50	Cyclopropane carboxylate	1000299-38-0	50.218	0.49
51	*n*-Hexadecanoic acid	57-10-3	50.842	0.34
52	Diethyl(1-aminocyclohexyl) phosphate	56372-35-1	51.444	2.26

The article "Extraction, Chemical Composition, and Protective Effect of Essential Oil from Chimonanthus nitens Oliv. Leaves on Dextran Sodium Sulfate-Induced Colitis in Mice" was published in 2022. Journal: Oxid Med Cell Longev.

## Data Availability

The (figures and tables) data used to support the findings of this study are included within the article.
